The article "Association between oral condition and subjective psychological well-being among older adults attending a university hospital dental clinic: A cross-sectional study" was published in 2023. Journal: PLoS One.

# Association between oral condition and subjective psychological well-being among older adults attending a university hospital dental clinic: A cross-sectional study

**DOI:** 10.1371/journal.pone.0295078

**Published:** 2023-11-28

**Authors:** Noriko Takeuchi, Nanami Sawada, Daisuke Ekuni, Manabu Morita

**Affiliations:** 1 Department of Preventive Dentistry, Okayama University Hospital, Okayama, Okayama, Japan; 2 Department of Preventive Dentistry, Graduate School of Medicine, Dentistry and Pharmaceutical Sciences, Okayama University, Okayama, Okayama, Japan; 3 Department of Oral Health, Takarazuka University of Medical and Health Care, Takarazuka, Hyogo, Japan; University of Minnesota School of Dentistry, UNITED STATES

## Abstract

Positive psychological well-being has a favorable impact on survival rates in both healthy and unhealthy populations. Oral health is also associated with psychological well-being, is multidimensional in nature, and includes physical, psychological, emotional, and social domains that are integral to overall health and well-being. This study aimed to identify the associations between individual and environmental characteristics, oral condition and nutritional status in relation to subjective well-being among older adults using the Wilson and Cleary conceptual model. The participants were older adults (age ≥ 60 years) attending a university hospital. Subjective well-being was assessed using the World Health Organization-5 Well-Being Index, oral condition was assessed based on the number of bacteria in the tongue coating, oral wettability, tongue pressure, occlusal force, oral diadochokinesis, and masticatory ability, and subjective swallowing function was assessed using the Eating Assessment Tool, number of remaining teeth, and number of functional teeth. In addition, factors related to well-being, including social networks, life–space mobility, nutritional status, smoking history, drinking history, and medical history were assessed. In the analysis, structural equation modeling was used to investigate the association between oral condition and subjective well-being. Confirmatory factor analysis revealed oral condition as a latent variable, including tongue pressure, oral diadochokinesis /pa/, /ta/, /ka/, occlusal force, masticatory ability, subjective swallowing function, and number of functional teeth. Structural Equation Modeling revealed that oral condition was positively correlated with nutritional status, and nutritional status was positively correlated with the World Health Organization-5 Well-Being Index. These findings suggest that oral condition may influence subjective well-being via nutritional status or social environmental factors.

The article "Association between oral condition and subjective psychological well-being among older adults attending a university hospital dental clinic: A cross-sectional study" was published in 2023. Journal: PLoS One.

## Introduction

Well-being is a positive state experienced by individuals and societies. Similar to health, it is a resource for daily life that is determined by social, economic, and environmental conditions [1]. The Geneva Charter for Well-being was endorsed at the Global Conference on Health Promotion in 2021, coordinated by the World Health Organization. It underlines the urgency of creating sustainable “well-being societies”.

In Japan, the average life expectancy is estimated to increase to 84.95 years for men and 91.35 years for women by 2065 [2]. As the ultimate goal of geriatrics is to achieve well-being, an important societal challenge is to identify factors related to subjective well-being to achieve a “100-year life period” among older adults [2].

Subjective well-being is defined as “all of the various types of evaluations, both positive and negative, that people make of their lives. It includes reflective cognitive evaluations, such as life satisfaction and work satisfaction, interest and engagement, and affective reactions to life events, such as joy and sadness” [3]. Positive psychological well-being is known to have a favorable impact on survival rates in both healthy and unhealthy populations [4]. Subjective well-being and health are closely associated with age [3, 4]. If older adults can maintain both subjective well-being and health commensurate with their age, they can extend their healthy life-span. On the other hand, poor subjective well-being has been reported to be associated with depression, functional limitations, low levels of wealth, unpaid work, a perceived lack of positive support from one’s spouse, children, and friends, a small social network [5, 6], smoking, low levels of physical activity, alcohol intake [7], and systemic disease such as stroke, chronic lung disease, rheumatoid arthritis, diabetes, and cancer [8].

Oral health is also known to be associated with psychological well-being. In a review by Peres et al. [9], oral health was defined as being multidimensional in nature and to include physical, psychological, emotional, and social domains, which are integral to overall health and well-being. In their scoping review, Badewy et al. [10] reported that poor oral health has a significant impact on the general health status of older adults. Appropriate interventions can also improve oral function among older adults [11]. Satisfaction with **diet** in everyday life has been shown to be associated with oral health-related quality of life (HRQoL) and subjective well-being in older Japanese adults, even after adjusting for a loss of teeth [12]. Occlusal force has been reported to be associated with psychological frailty in Japanese community-dwelling older adults [13] considering the possibility that reduced nutritional intake and appetite may mediate the relationship between occlusal force and psychological frailty. The complete loss of teeth has been associated with deteriorations in psychological and subjective well-being in older adults [14], based on the fact that tooth loss leads to a loss of facial aesthetics and personality, which affects the individual’s social performance and ability to form social relationships, resulting in low levels of well-being.

The article "Association between oral condition and subjective psychological well-being among older adults attending a university hospital dental clinic: A cross-sectional study" was published in 2023. Journal: PLoS One.

Wilson and Cleary [15] developed a model that clearly conceptualizes the relationship between clinical factors and HRQoL. Their model describes the causal pathways of several determinants in HRQoL, including biological and physiological factors such as cellular function and organs, symptom status (i.e., patients’ perceptions of cognitive, physical, and emotional functioning), functional health (i.e., physical, psychological, social, and role functioning), general health perceptions (i.e., subjective evaluation of the integrated concept of all health aspects), and overall quality of life (i.e., subjective evaluation of the patients’ overall well-being). In the dental field, this model has been used to link xerostomia, edentulism, and the need for prosthodontic treatment to oral health-related QoL (OHRQoL) among older adults [16–20]. These previous studies support part of the key direct pathways hypothesized by Wilson and Cleary [15]. However, the findings were limited to edentulous older people with dentures [17], xerostomia [18], or only a few diagnostic items for oral health status [16, 18, 19]; few reports have examined psychosocial factors [16, 19].

Therefore, we hypothesized that the oral condition may be associated with subjective well-being among older adults even when considered alongside nutritional status and both individual and environmental characteristics.

Given this background, the present study aimed to identify the associations between individual and environmental characteristics, oral condition, and nutritional status in relation to subjective well-being among older adults using the Wilson and Cleary conceptual model (Fig 1). The specific aim was to determine how nutritional status and environmental characteristics are associated with the effects of various oral conditions on subjective well-being among older adults.

**Fig 1:** Hypothetical model using the Wilson and Cleary conceptual model. Path coefficients and p-values are shown above. Rectangles indicate observed variables, and ovals show latent variables. Abbreviations: ODK, oral diadochokinesis; EAT-10, the 10-item Eating Assessment Tool; MNA, Mini-Nutritional Assessment; LSNS, Lubben Social Network Scale; LSA, Life Space Assessment; WHO-5, World Health Organization-5 Well- Being Index.

The article "Association between oral condition and subjective psychological well-being among older adults attending a university hospital dental clinic: A cross-sectional study" was published in 2023. Journal: PLoS One.

## Materials and methods

### Study participants

The participants in this cross-sectional study were older patients (age ≥ 60 years) who had regularly visited the Preventive Dentistry Clinic at Okayama University Hospital from November 2017, when recruitment began, to January 2019. Those who could not respond to the questionnaire or walk independently were excluded. Written, informed consent to participate in this study was obtained from all participants. We had no access to information that could identify individual participants during or after data collection. This study followed the STROBE guidelines regarding cross-sectional studies.

### Evaluation of subjective psychological well-being

In this study, the World Health Organization-5 Well-Being Index (WHO-5), which is composed of five items that measure positive mood, vitality, and general interests [21, 22], was used to assess subjective well-being. The Japanese version of the WHO-5 has been shown to be reliable and valid in older adults [21]. In the WHO-5, the respondents are asked to rate their subjective well-being in the previous 2 weeks on a 6-point Likert scale from 0 (not present) to 5 (constantly present). The total raw score is then multiplied by 4 to obtain the final score, with higher scores indicating greater psychological well-being [23].

### Assessment of oral condition

After calibration, three trained dentists assessed the participants’ oral condition based on the number of remaining teeth [13], the number of functional teeth, and the following seven items recommended by the Japanese Society of Gerontology [24] as diagnostic items for oral hypofunction: number of bacteria in the tongue coating, oral wetness, tongue pressure, occlusal force, oral diadochokinesis (ODK), masticatory ability, and swallowing function.

#### Number of bacteria in tongue coating

To collect samples for counting the number of bacteria in the tongue coating, the central part of the tongue was swabbed three times with a sterile cotton swab over a length of 1 cm [24–26]. A constant-pressure device was used to reduce the variation in operator performance [27]. Next, a bacterial counter (Panasonic Healthcare, Tokyo, Japan) was used to measure the number of bacteria in 1 mL of collected sample. Samples were taken twice, and then the average of the two samples was calculated.

#### Oral wetness

To measure the degree of oral wetness, an oral moisture checker (Mucus®; Life Co., Saitama, Japan) [24–26] was used on the center of the dorsum of the tongue at a distance of 1 cm from the tip of the tongue and the right and left buccal mucosa. After attaching a special sensor cover, the sensor was pressed with a force of approximately 200 g to achieve uniform contact with the test surface. This was held for about 2 seconds until the device displayed the measured value. Measurements were performed twice, and oral wetness was defined as the average value for all measurements.

The article "Association between oral condition and subjective psychological well-being among older adults attending a university hospital dental clinic: A cross-sectional study" was published in 2023. Journal: PLoS One.

#### Tongue pressure

A tongue depressor (TPM-01; JMS, Hiroshima, Japan) [24–26, 28, 29] was used to measure tongue pressure. In this study, we defined the maximum tongue pressure as the pressure generated when the balloon of the tongue depressor probe was arbitrarily crushed between the tongue and palate on the anterior surface of the palate and held for several seconds at maximum force. Measurements were performed with dentures, if present, practiced beforehand, and carried out twice with a rest in between. Finally, the average value from all measurements was calculated.

#### Occlusal force

An occlusal diagnostic system consisting of a pressure-sensitive film (Dental Prescale® II; Fujifilm, Kuala Lumpur, Malaysia) and a pre-calibrated scanner (GT-X830; Seiko Epson, Suwa, Japan) [24–26, 30, 31] was used to measure occlusal force. All participants were asked to bite the pressure-sensitive film with maximum force for 3 seconds. Denture wearers underwent the measurement with their dentures in place. Measurements were performed only once.

#### Oral diadochokinesis (ODK)

The speed and elaboration of tongue and lip movements were assessed based on ODK [24–26, 32, 33]. In this study, we measured /pa/, /ta/, and /ka/ sounds, which can be used to evaluate lip, anterior tongue, and posterior tongue movements, respectively. All participants were instructed to repeat each sound as quickly as possible for 5 seconds. The number of pronunciations was recorded using a digital counter (Kenko-kun® Handy; Takei Scientific Instruments, Niigata, Japan), after which, the number of pronunciations per second was calculated. Each sound pronunciation was measured twice, and then the average value was calculated.

#### Masticatory ability

To assess masticatory ability, the glucose concentration after chewing gummy jelly (Glucolumn®; GC, Tokyo, Japan) for 20 seconds was measured [24–26]. After chewing, the participants were instructed to hold 10 mL of water in their mouths before draining it into a filtration mesh. A glucose sensor (Glucosensor® GS-II; GC) was then used to measure the glucose concentration in the filtrate. Each measurement was performed twice, and then the average value was calculated.

#### Swallowing function

To assess swallowing function, we administered the Japanese version of the Eating Assessment Tool (EAT-10) (Nestlé, Vevey, Switzerland) [24–26, 34, 35], which is a self-administered questionnaire composed of 10 questions on swallowing. Each question is scored from 0 to 4, with the total score ranging between 0 and 40, and a lower total score indicating fewer swallowing problems.

The article "Association between oral condition and subjective psychological well-being among older adults attending a university hospital dental clinic: A cross-sectional study" was published in 2023. Journal: PLoS One.

#### Numbers of teeth present and number of functional teeth

The oral examinations involved counting the number of remaining teeth and the number of functional teeth. The number of functional teeth was defined as the sum of the number of natural teeth present and prostheses (e.g., pontics, implants, dentures) replacing any missing teeth. Stump teeth and those with severe decay were not considered [25, 26, 36].

### Questionnaire survey

#### Social network

To assess each participant’s relationships with others and the community, we administered the abbreviated version of the Lubben Social Network Scale (LSNS-6) [37]. The original LSNS is a social network scale for older adults developed by Lubben in 1988 [38]. The Japanese version of the LSNS-6 has been shown to be reliable and valid [39]. The LSNS-6 is composed of three questions that assess kinship relationships (“How many relatives do you see or keep in touch with at least once a month?”, “How many relatives do you see or talk to at least once a month?”, and “How many relatives do you feel free to talk to about your private matters?”), and three similar questions that assess non-kinship relationships. The three kinship items are repeated for connections with people other than relatives, except the word “relatives” is replaced with “friends”. The score for the entire scale is an equally weighted version of the six items, with the total score ranging from 0 to 30.

#### Life–space mobility (LSM)

LSM, which is associated with nutritional status [40], social networks [41], and tongue pressure [42], was measured using the life–space assessment (LSA). This assessment quantifies movement during the last month into five life–space levels. Specific questions on the LSA are: “During the past 4 weeks, have you been to: [Level 1] ‘other rooms of your home besides the room where you sleep?’, [Level 2] ‘an area outside your home, such as your porch, deck, patio, hallway (of an apartment building), garage, or in your own yard or driveway?’, [Level 3] ‘places in your neighborhood other than your own yard or apartment building?’, [Level 4] ‘places outside your neighborhood but within your own town?’, and [Level 5] ‘places outside your town?’” For each level, participants are asked how often they traveled to that area and whether they required equipment (e.g., a walker) or the assistance of another person to access that space. The life–space score is the sum of the score for each of the five levels. Individual level scores were obtained by multiplying the level number (1–5), a value for the frequency (1 = less than once per week, 2 = 1–3 times/week, 3 = 4–6 times/week, 4 = daily), and a value for independence (2 = no assistance, 1.5 = use of equipment only, 1 = assistance from another person with or without equipment). The life–space score ranges from 0 (never leaves one’s bedroom) to 120 (able to move around outside of town daily without assistance). The LSA has been translated in to Japanese by the Physical Therapy Association [43] and is used for older adults in Japan [44].

The article "Association between oral condition and subjective psychological well-being among older adults attending a university hospital dental clinic: A cross-sectional study" was published in 2023. Journal: PLoS One.

#### Nutritional status

Nutritional status was assessed using the Mini-Nutritional Assessment (MNA; Nestlé) [45]. The MNA is a nutrition screening tool specifically designed for older adults [46] and is widely used in Japan [26, 47, 48]. The MNA is a 30-point scale composed of 18 items that assess four aspects of nutritional status: an anthropometric assessment (body mass index, weight loss, upper middle arm circumference, and calf circumference), a global assessment (mobility, prescription medications, independent living, psychological stress or acute disability, pressure ulcers or bedsores, and neuropsychological problems), a dietary assessment (complete daily diet, decreased dietary intake, fluid intake, protein intake, fruit and vegetable intake, and feeding methods), and self-assessment (nutritional status and health status) [49]. The higher the total score, the better the nutritional status.

#### Smoking and alcohol history

Smoking and alcohol histories were confirmed by a questionnaire. Smoking history was categorized into two groups: never smokers and a combination of current and former smokers [25]. For alcohol history, the respondents were asked to indicate how much beer, sake, shochu, whiskey, or wine they each drank per day. The amount of ethanol was calculated in grams as follows: 633 mL beer contains 23 g of ethanol, 180 mL sake contains 23 g of ethanol, 180 mL shochu contains 36 g of ethanol, 30 mL whiskey contains 10 g of ethanol, and 60 mL wine contains 9 g ethanol [50]. Heavy drinking was defined as ethanol intake of 22 g/day or more [51].

#### Medical information

A questionnaire composed of items on the following conditions that have been linked to well-being was used to record medical history: stroke, chronic lung diseases, rheumatoid arthritis, diabetes, and cancer [8]. Responders who indicated that they were “currently receiving treatment” for any of the disease were classified as having that disease.

The article "Association between oral condition and subjective psychological well-being among older adults attending a university hospital dental clinic: A cross-sectional study" was published in 2023. Journal: PLoS One.

### Statistical analysis

Intra- and inter-examiner reliability were investigated using intraclass correlation coefficients (ICCs). ICC values > 0.75 were considered indicative for excellent stability, 0.40–0.75 for fair to good stability, and < 0.40 for poor stability [52]. Descriptive statistics were conducted for demographic status, subjective psychological well-being, oral conditions, social status, nutritional status, and medical information. Fig 1 shows the hypothetical model with reference to previous studies [13, 40–42] using the Wilson and Cleary conceptual model. Structural equation modeling (SEM) was applied to analyze the relationship between oral condition and subjective psychological well-being. The first step was to examine the components of oral condition using confirmatory factor analysis (CFA). Next, the hypothetical model was examined. Based on previous research, the affect from oral condition to environmental characteristics was also examined. The association between oral condition and subjective psychological well-being was then analyzed using Spearman’s correlation coefficient. Maximum likelihood estimation considering missing data was performed in the SEM. The comparative fit index (CFI), Tucker–Lewis index (TLI), and root mean square error of approximation (RMSEA) were reported. The acceptable fit index criteria used in the SEM were as follows: CFI > 0.90, TLI > 0.90, and RMSEA < 0.10. Stata Version 17.0 software (Stata Corp LLC, College Station, TX) was used for all analyses with the significance level set at 0.05.

### Ethical considerations

This study was conducted in accordance with the tenets of the Declaration of Helsinki, and all procedures involving human participants were approved by the ethics committee of Okayama University Graduate School of Medicine, Dentistry and Pharmaceutical Sciences and Okayama University Hospital (approval No.: 1803–038).

## Results

In total, 218 participants were analyzed in this study (male: n = 66 [30.3%], female: n = 152 [69.7%]; mean age: 75.0 years). The ICCs for the intra- and inter-examiner reliability were 0.984 (95% Confidence Interval [CI]: 0.934–0.996) and 0.985 (95% CI: 0.940–0.998), respectively. The characteristics of the participants are shown in Table 1. Descriptive statistics of the univariate associations between oral condition and well-being are presented in Table 2.

**Table 1:** The characteristics of the participants.

	Total	Male	Female
	(n = 218)	(n = 66)	(n = 152)
Age (years)	75.0 ± 6.8^a^	75.5 ± 6.8	74.8 ± 6.8
WHO-5	68.3 ± 18.6	89.5 ± 18.5	68.1 ± 18.7
Number of bacteria in tongue coating (CFU × 106/mL)	18.8 ± 17.6	21.0 ± 19.4	17.9 ± 16.7
Oral wetness	29.0 ± 2.0	28.8 ± 2.2	29.1 ± 2.0
Tongue pressure (kPa)	31.3 ± 8.4	31.1 ± 8.8	31.4 ± 8.2
Occlusal force (N)	528.9 ± 384.2	652.8 ± 446.1	485.1 ± 351.1
ODK (times/s)			
/pa/ sound	5.9 ± 0.9	5.8 ± 0.9	5.9 ± 0.8
/ta/ sound	5.9 ± 0.8	5.9 ± 0.9	5.9 ± 0.8
/ka/ sound	5.6 ± 0.8	5.4 ± 1.0	5.7 ± 0.8
Masticatory ability (mg/dL)	172.1 ± 67.7	178.8 ± 69.5	169.5 ± 67.0
EAT-10	0.9 ± 2.6	1.0 ± 3.4	0.9 ± 2.2
Number of remaining teeth	20.2 ± 7.0	20.1 ± 7.6	20.3 ± 6.7
Number of functional teeth	26.3 ± 3.4	26.2 ± 3.3	26.4 ± 3.5
LSNS-6	15.3 ± 5.8	16.2 ± 6.7	14.9 ± 5.4
LSA	92.1 ± 24.2	93.5 ± 24.7	91.4 ± 24.0
MNA	25.1 ± 2.6	25.5 ± 2.5	24.9 ± 2.7
Smoking experience	7 (3.2)^b^	4 (6.1)	3 (2.0)
Heavy drinking	37 (30.0)	4 (36.9)	13 (8.6)
Stroke	5 (2.3)	3 (4.5)	2 (1.3)
Chronic lung diseases	7 (3.2)	1 (1.5)	6 (3.9)
Rheumatoid arthritis	5 (2.3)	0 (0.0)	5 (3.3)
Diabetes	25 (11.4)	7 (10.6)	18 (11.8)
Cancer	3 (1.4)	1 (1.5)	2 (1.3)

^a^ average ± standard deviation

^b^ n (%)

Abbreviations: WHO-5, the World Health Organization-5 Well-Being Index; ODK, Oral diadochokinesis; EAT-10, the Eating Assessment Tool; LSNS-6, the Lubben Social Network Scale, LSA, life–space assessment; MNA, the Mini-Nutritional Assessment

The article "Association between oral condition and subjective psychological well-being among older adults attending a university hospital dental clinic: A cross-sectional study" was published in 2023. Journal: PLoS One.

**Table 2:** Descriptive statistics for the univariable association between oral condition and the WHO-5.

	Coefficient	P-value^a^
Number of bacteria in tongue coating (CFU × 106/mL)	0.060	0.382
Oral wetness	0.026	0.697
Tongue pressure (kPa)	0.021	0.760
Occlusal force (N)	0.026	0.719
ODK (times/s)		
/pa/ sound	0.060	0.375
/ta/ sound	0.038	0.579
/ka/ sound	0.026	0.700
Masticatory ability (mg/dL)	0.055	0.417
EAT-10	-0.178	0.008
Number of remaining teeth	0.023	0.736
Number of functional teeth	-0.060	0.379

^a^ Spearman’s correlation coefficient

Abbreviations: ODK, Oral diadochokinesis; EAT-10, the Eating Assessment Tool

The multicollinearity of each index of oral condition was confirmed. the Variance Inflation Factor ranged from 1.03 to 3.36, so all indexes were used in the analysis. The results using all diagnostic items of the hypothetical model (Fig 1) were accepted by STATA, and no notification messages were obtained about analyzed parameters. CFA was conducted on oral condition and individual characteristics. Even after excluding the number of bacteria in the tongue coating, oral wetness, and the number of remaining teeth, which showed p > 0.05 for the latent variable oral condition, the model fit was poor (RMSEA = 0.096, CFI = 0.903, TLI = 0.864). Specification of residual correlations between masticatory ability and occlusal force (modification index [MI] = 18.783, standardized expected parameter change [EPC] = 0.310), masticatory ability and number of functional teeth (MI = 12.556, standardized EPC = 0.243), and ODK /ka/ sound, and number of functional teeth (MI = 6.778, standardized EPC = 0.200) improved the model fit.

The article "Association between oral condition and subjective psychological well-being among older adults attending a university hospital dental clinic: A cross-sectional study" was published in 2023. Journal: PLoS One.

SEM in the hypothetical model was performed using the modified oral condition and individual characteristics. After removing paths with p > 0.05, all path coefficients were statistically significant and showed a good fit (RMSEA = 0.042, CFI = 0.963, TLI = 0.949) (Fig 2). SEM revealed that oral condition was significantly associated with MNA score (standardized path coefficient = 0.160, p = 0.036). The MNA score was significantly associated with the WHO-5 score (standardized path coefficient = 0.190, p = 0.018). Environmental characteristics were significantly associated with oral condition (standardized path coefficient = 0.223, p = 0.027), MNA score (standardized path coefficient = 0.351, p = 0.001), and WHO-5 score (standardized path coefficient = 0.361, p <0.001). When the path way from oral condition to environmental characteristics was examined (Fig 2), each path was significant (p < 0.05) and the goodness of fit was adequate (RMSEA = 0.042, CFI = 0.963, TLI = 0.949).

**Fig 2:** Structural equation modeling of the relationship between oral condition and subjective well-being (final model). Path coefficients and p-values are shown above. Rectangles indicate observed variables, and ovals show latent variables. Values of single-headed arrows indicate standardized coefficients. The levels of significance considered were *p < 0.05, **p < 0.01, and ***p < 0.001. Abbreviations: ODK, oral diadochokinesis; EAT-10, the 10-item Eating Assessment Tool; MNA, Mini-Nutritional Assessment; LSNS, Lubben Social Network Scale; LSA, Life–Space Assessment; WHO-5, World Health Organization-5 Well- Being Index.

## Discussion

The results of this study revealed that oral condition was not directly associated with well-being, but was associated with nutritional status, and that nutritional status was associated with well-being.

The association observed between oral condition and nutrition is supported by previous studies [53, 54]. In a systematic review and meta-analysis, Toniazzo et al. [53] reported that subjects with good nutritional status had a significantly higher number of tooth pairs/(functional teeth units) than did those at risk for malnutrition and those with poor nutrition. In another review, Iwasaki et al. [54] reported a study that supported a possible relationship between poor oral function and inadequate, poor-quality diets and malnutrition. They found that older adults with poor oral function were more likely to have low dietary intake and poor nutritional status, and that malnourished older adults were more likely to have poor oral function.

The article "Association between oral condition and subjective psychological well-being among older adults attending a university hospital dental clinic: A cross-sectional study" was published in 2023. Journal: PLoS One.

Previous studies have also shown that nutrition affects well-being. A systematic review of randomized controlled trials [55] reported that the protein and amino acids found in beef may positively influence well-being through improved physical function in healthy adults aged ≥ 50 years. Piqueras et al. [56] examined the relationship between subjective well-being and healthy lifestyle in young adults and found that eating lunch, fruits, and vegetables every day was associated with good well-being. Obesity has been reported to be associated with depression. Therefore, they considered that the daily intake of lunch, fruits, and vegetables contributes to well-being because it limits fat intake and prevents obesity [57]. In the present study, nutritional status may have been related to well-being through physical function improvement and obesity prevention.

This study showed pathways from environmental characteristics to oral health and from oral health to environmental characteristics. Previous studies [58–60] have suggested that poor social support and poor social networks adversely affect dental caries, gingivitis, and tooth loss. Those studies further indicated that social capital is commonly associated with psychological distress, which may increase the risk of periodontal disease and lead to increased smoking and consumption of sweets, which in turn, may increase the risk of dental caries and periodontal disease. Moreover, individuals who have poor chewing skills or difficulty with verbal and emotional communication due to poor oral health may experience a decrease in self-confidence, which predisposes them to loneliness [5]. The findings of this study also suggest that there may be a bidirectional association between oral condition and environmental characteristics.

In this study, environmental characteristics were associated with nutritional status. Ingham et al. [61] reported that the low support for social environment profile had the poorest nutritional status. Mills et al. [62] reported that individuals with restricted social networks had lower nutrition risk scores. They discussed that close relationships may increase opportunities to share meals and resources for food-related activities such as grocery shopping and meal preparation, and that eating with others has been shown to improve food intake and reduce nutritional risks.

In the present study, an association was observed between social networks and well-being. Becker et al. [63] reported that parenthood, marital status, and social networks are related to the well-being and mental health of older people. Buckley et al. [64] investigated the association between the LSNS-6 and subjective health in older adults in Puerto Rico and found that connections with friends affect subjective health through a psychological sense of community. These previous results support the findings of the present study.

The article "Association between oral condition and subjective psychological well-being among older adults attending a university hospital dental clinic: A cross-sectional study" was published in 2023. Journal: PLoS One.

The neuromuscular units of the face and oral cavity are involved in speech, chewing and swallowing. Decremental changes occur in these motor units and their coordinated functions during the aging process. To measure events per unit time, ODK tests the ability to make articulatory speech and antagonistic movements in quick succession, alternating opposing muscle groups [33]. This ability is typically evaluated by measuring how fast an individual can repeat the monosyllabic sounds /pa/, /ta/, and /ka/, which in turn, allows for an assessment of the motor ability of the lips, as well as of the anterior and posterior sections of the tongue. While the concept of ODK has been predominantly reported in Japan, additional studies have been conducted in other regions [32, 33, 65]. Previous studies have shown that ODK has high test–retest reliability [66, 67]. The validity of ODK as an index for assessing oral function in older adults has also been reported by various studies [36, 68].

### Limitations

This study did have some limitations. First, as this was a cross-sectional study, it was not possible to establish a causal relationship between each factor. Therefore, further longitudinal studies are needed. Second, we did not examine some of the environmental characteristics that have previously been reported to be related to well-being (e.g., low wealth, unpaid work). Third, the study participants were relatively healthy older patients who regularly visited the university hospital. It is possible that direct associations were not shown as being statistically significant. Therefore, the generalizability of the findings is limited. Further studies with a larger patient population are warranted.

## Conclusions

The results of the present study suggest associations between oral condition and nutritional status and between nutritional status and subjective well-being among older adults attending a university hospital dental clinic, as influenced by environmental characteristics. Oral condition may influence subjective well-being through nutritional status.

## Supporting information

S1 Dataset (XLSX)
